The article "Efficacy of Apatinib plus S-1 Therapy in the Treatment of Advanced Gastric Cancer Patients and the Effect on the Levels of Tumor Markers and Th1 and Th2-Like Cytokines" was retracted in 2023. Reasons: signs of a paper mill; compromised peer review; unreliable results or conclusions.

# Efficacy of Apatinib plus S-1 Therapy in the Treatment of Advanced Gastric Cancer Patients and the Effect on the Levels of Tumor Markers and Th1 and Th2-Like Cytokines

**DOI:** 10.1155/2022/8060026

**Published:** 2022-04-27

**Authors:** Jishu Gu, Xuejiao Ni, Jinfeng Ji, Guohua Wei, Lei Shi, Chunming Xu

**Affiliations:** Affiliated Tumor Hospital of Nantong University, Nantong, Jiangsu 226006, China

## Abstract

**Objective:**

To assess the efficacy of apatinib plus S-1 therapy in the treatment of advanced gastric cancer patients and the effect on the levels of tumor markers and Th1 and Th2-like cytokines.

**Methods:**

From October 2019 to December 2020, 100 patients with advanced gastric cancer assessed for eligibility were recruited and assigned at a ratio of 1 : 1 to receive either S-1 regimen (tegafur, gimeracil, and oteracil potassium capsules) (observation group) or apatinib plus S-1 therapy (experimental group). Outcome measures included clinical efficacy serum tumor marker levels, Th1 and Th2-like cytokine levels, time to progression (TTP), overall survival (OS), and adverse events.

**Results:**

The S-1 therapy plus apatinib was associated with a significantly higher efficacy versus S-1 therapy alone (*P* < 0.05). The eligible patients given S-1 therapy plus apatinib showed significantly lower levels of serum carcinoembryonic antigen (CEA), glycoantigen 199 (CA199), and glycoantigen 125 (CA125) versus those receiving S-1 therapy (*P* < 0.05). S-1 therapy plus apatinib outperformed the single therapy of S-1 therapy in mitigating the levels of interferon-*γ* (IFN-*γ*), tumor necrosis factor-*α* (TNF-*α*), interleukin-4 (IL-4), and interleukin-10 (IL-10) (*P* < 0.05). There was no statistically significant difference in the incidence of adverse reactions between the two groups (*P* > 0.05). S-1 therapy plus apatinib was associated with a significantly shorter TTP (5.2 ± 0.7 months) and a longer OS (9.3 ± 2.5 months) versus S-1 therapy alone (7.1 ± 1.3, 5.1 ± 1.3 months) (*P* < 0.05).

**Conclusion:**

The efficacy of apatinib plus S-1 therapy showed better improvement in lowering the serum tumor marker levels and ameliorating the Th1 and Th2-like cytokine levels versus S-1 therapy alone, so it is worthy of clinical application.

## 1. Introduction

Gastric cancer is a common malignant tumor in the digestive system that originates from the micromucosal epithelium, with the highest incidence among all malignant tumors in China [1]. Gastric cancer is mostly triggered by *Helicobacter pylori* infection, and most cases have progressed to the advanced stage by the time of diagnosis due to the insidiousness of its symptoms at the early stage [2]. Surgery is considered ineffective for patients with advanced gastric cancer, so chemotherapy is mostly performed to inhibit tumor development and prolong the survival of patients [3]. S-1 therapy is a fluorouracil derivative oral anticancer agent and is commonly used in second-line chemotherapy for gastric cancer. Relevant research has revealed pronounced side effects of S-1 therapy, for which patients are mostly intolerant [4], and monotherapy is inconsistent with the principle of combined chemotherapy for malignancies treatment [5]. At present, there are extensive clinical studies showing a close association between vascular endothelial growth factor and tumorigenesis and development [6]. Apatinib inhibits neoangiogenesis in tumor tissue, which can prolong the survival of patients with advanced gastric cancer [7]. Serum tumor markers serve to determine tumor severity and prognosis, and common serum tumor markers include carcinoembryonic antigen (CEA), glycoantigen 199 (CA199), and glycoantigen 125 (CA125) [8]. Clinical research has shown that Th1 and Th2-like cytokines regulate immune function, and trauma may lead to immune imbalance due to abnormal Th1 and Th2-like cytokines levels [9]. Accordingly, the present study recruited 100 patients with advanced gastric cancer between October 2019 and December 2020 to assess the efficacy of apatinib plus S-1 therapy in the treatment of advanced gastric cancer patients and the effect on the levels of tumor markers, Th1 and Th2-like cytokines.

The article "Efficacy of Apatinib plus S-1 Therapy in the Treatment of Advanced Gastric Cancer Patients and the Effect on the Levels of Tumor Markers and Th1 and Th2-Like Cytokines" was retracted in 2023. Reasons: signs of a paper mill; compromised peer review; unreliable results or conclusions.

## 2. Materials and Methods

### 2.1. Baseline Data

From October 2019 to December 2020, 100 patients with advanced gastric cancer assessed for eligibility were recruited and assigned at a ratio of 1 : 1 to an observation group or an experimental group. The patients in the observation group were aged 35–77 years with a duration of disease of 2–6 years, and the patients in the experimental group were aged 36–78 years with a duration of disease of 2–7 years. The studies involving human participants were reviewed and approved by our hospital (no. NT2937). The patients provided their written informed consent to participate in this study.

### 2.2. Inclusion and Exclusion Criteria

Inclusion criteria were as follows: patients met the clinical diagnosis criteria of gastric cancer, with a Karnofsky Performance Scale (KPS) score of ≥60 points, and with an expected survival of ≥3 months.

Exclusion criteria were as follows: patients with severe heart, liver, kidney, and other organ dysfunction, with other systemic tumor diseases, with cognitive impairment, with contraindications to chemotherapy, and with an allergy to the ingredients of the drugs used.

## 3. Methods

Patients in both groups were treated with conventional therapy, including acid suppression, antiemetic, hepatoprotection, and renal protection. The patients in the observation group were treated with S-1 therapy (Qilu Pharmaceutical Co., Ltd., State Pharmacopoeia H20100151, tegafur 25 mg, gimeracil 7.25 mg, and oteracil potassium 24.5 mg), and the baseline amount of the first dose for adults was 60 mg/time for body surface area >1.5 m^2^, 50 mg/time for body surface area 1.25–1.5 m^2^, and 40 mg/time for body surface area <1.25 m^2^, 2 times/d, 30 min after breakfast and dinner, and the medication was performed continuously for 14 d, after which the medication was stopped for 14 d, with 28 d as a course of treatment. The patients in the experimental group were given apatinib mesylate tablets (Jiangsu Hengrui Medicine Co., Ltd., State Drug Administration H20140103, 0.25 g) in addition to S-1 therapy. The initial dose of 500 mg was given orally, and the dose was gradually increased to 850 mg once/d based on the patient's tolerance, with 28 d as a course of treatment.

The article "Efficacy of Apatinib plus S-1 Therapy in the Treatment of Advanced Gastric Cancer Patients and the Effect on the Levels of Tumor Markers and Th1 and Th2-Like Cytokines" was retracted in 2023. Reasons: signs of a paper mill; compromised peer review; unreliable results or conclusions.

### 3.1. Endpoints

1. Clinical efficacy was evaluated via upper abdominal computed tomography (CT) scanning: complete remission (CR): tumor disappeared for more than 1 month and no new lesions were found; partial remission (PR): tumor lesions decreased in volume ≥30% and no new lesions were found; stable disease (SD): tumor volume decreased <30% with stable symptoms; progressive disease (PD): new lesions were found and tumor volume increased by more than 20%. Total efficacy = (number of CR cases + number of PR cases)/total number of cases × 100%.
2. Serum tumor marker levels: serum tumor markers including serum CEA, CA199, and CA125 were determined by electrochemiluminescence immunoassay. The kits were purchased from Roche, USA, and the equipment instrument used was Hitachi ElecSys 2010 fully automated electrochemiluminescence instrument, purchased from Hitachi, Japan, which was operated in strict accordance with the kit instructions.
3. Th1 and Th2-like cytokine levels: Th1 and Th2-like cytokines, including *γ*-interferon (IFN-*γ*), tumor necrosis factor-*α* (TNF-*α*), interleukin-4 (IL-4), and interleukin-10 (IL-10), were determined by ELISA, and the kits were purchased from Shanghai Baili Biotechnology Co., Ltd. and were operated in strict accordance with the kit instructions.
4. Time to progression (TTP) and overall survival (OS): TTP refers to the time from the beginning of chemotherapy to tumor progression, and OS refers to the time from the beginning of chemotherapy to the final follow-up or death. TTP and OS of the patients were recorded for comparison. Toxic effects were observed and recorded according to the toxicity manifestation and grading criteria established by the National Cancer Institute (NCL). The follow-up period is 1 year, with a closing date of December 31, 2021.

The article "Efficacy of Apatinib plus S-1 Therapy in the Treatment of Advanced Gastric Cancer Patients and the Effect on the Levels of Tumor Markers and Th1 and Th2-Like Cytokines" was retracted in 2023. Reasons: signs of a paper mill; compromised peer review; unreliable results or conclusions.

### 3.2. Statistical Analysis

SPSS 22.0 software was used for data analyses. The count data were expressed as (*n* (%)) and processed using the chi-square test, and the measurement data were expressed as ($\bar{\text{x}}$ ± *s*) and processed using the *t*-test. Differences were considered statistically significant at *P* < 0.05.

## 4. Results

### 4.1. Baseline Data

The two groups showed similar baseline data (*P* > 0.05) (Table 1).

### 4.2. Clinical Efficacy

The S-1 therapy plus apatinib was associated with a significantly higher efficacy versus S-1 therapy alone (*P* < 0.05) (Table 2).

### 4.3. Serum Tumor Marker Levels

The eligible patients given S-1 therapy plus apatinib showed significantly lower levels of serum CEA, CA199, and CA125 versus those receiving S-1 therapy (*P* < 0.05) (Table 3).

### 4.4. Th1 and Th2-Like Cytokine Levels

S-1 therapy plus apatinib outperformed the single therapy of S-1 therapy in mitigating the levels of IFN-*γ*, TNF-*α*, IL-4, and IL-10 (*P* < 0.05) (Table 4).

### 4.5. Adverse Event and Survival

There was no statistically significant difference in the incidence of adverse reactions between the two groups (*P* > 0.05). S-1 therapy plus apatinib was associated with a significantly shorter TTP (5.2 ± 0.7 months) and a longer OS (9.3 ± 2.5 months) versus S-1 therapy alone (7.1 ± 1.3, 5.1 ± 1.3 months) (*P* < 0.05) (Table 5).

## 5. Discussion

Chemotherapy is a common clinical treatment for patients with advanced gastric cancer, which prolongs the survival and improves the quality of life of patients [10]. Combination chemotherapy with multiple drugs is currently the main regimen of chemotherapy for patients with advanced gastric cancer and is divided into first-line chemotherapy, second-line chemotherapy, and third-line chemotherapy [11]. Drugs for first-line chemotherapy mostly include fluorouracil, platinum, and anthracyclines, but the poor physical condition of patients frequently accompanied by anemia at this stage may result in intolerance to the first-line chemotherapy regimen [12]. In recent years, new chemotherapeutic drugs have gained clinical recognition for their promising efficacy in patients with advanced gastric cancer. S-1 is a new generation of fluorouracil oral drugs made of tegafur, gimeracil, and oteracil potassium. It significantly increases the concentration of fluorouracil in patients' blood and tumor cells with a long half-life and long-lasting efficacy, which is considered more stable than traditional fluorouracil drugs. In addition, S-1 protects the mucosa of the digestive tract and can effectively reduce adverse gastrointestinal reactions, thereby improving the tolerability of patients with advanced gastric cancer. Extensive clinical studies have shown that the S-1 therapy can achieve similar therapeutic effects and higher clinical safety versus the fluorouracil treatment regimen for advanced gastric cancer [13]. Apatinib is a new antitumor angiogenic drug that competitively binds to tyrosine ATP binding sites within VEGFR-2 to interfere with VEGF signaling, and it also inhibits platelet production factor receptor *β* and c-kit, thereby compromising tumor angiogenesis. Apatinib is excreted through the intestine in a short time, and the residual amount in the body after 4 d of discontinuation remains only about 22.5%, indicating a high safety profile [14]. Phase I and II clinical trials found that the disease-free progression and overall survival were significantly prolonged in patients with advanced gastric cancer who failed second-line chemotherapy and were switched to apatinib. The State Food and Drug Administration has also included apatinib in the third-line and higher treatment regimens for advanced gastric cancer [15].

The article "Efficacy of Apatinib plus S-1 Therapy in the Treatment of Advanced Gastric Cancer Patients and the Effect on the Levels of Tumor Markers and Th1 and Th2-Like Cytokines" was retracted in 2023. Reasons: signs of a paper mill; compromised peer review; unreliable results or conclusions.

The vascular endothelial growth factor (VEGF) induces tumor angiogenesis, which promotes tumor invasion and metastasis. Apatinib is a novel small molecule tyrosine kinase inhibitor of the vascular endothelial growth factor receptor (VEGFR-2) that competitively binds to the receptor intracellular tyrosine F6 site and highly selectively inhibits VEGFR-2 enzymatic activity, thus blocking the signal transduction pathway after VEGFR binding to VEGFR-2 and inhibiting tumor vascular production [8]. A clinical study has shown that the basic control rate of apatinib for advanced gastric cancer can reach 42% [9]. It can respond to the normal function of mitochondria in tumor cells and induce apoptosis and differentiation of tumor cells. Combined with tegafur, it contributes to the enhancement of the body's immune surveillance and clearance of mutated cells, accelerates the self-repair of gastric mucosal epithelial cells, and thus promotes the dominant expression of Th1-like immune cytokines, as well as downregulates the levels of Th2-like cytokines [15]. The present study showed that the S-1 therapy plus apatinib was associated with a significantly higher efficacy versus S-1 therapy alone, indicating a better treatment efficiency after the application of apatinib. CEA is a glycoprotein that is produced by colorectal cancer tissue and is one of the spectral antitumor markers [16], and both CA199 and CA125 are glycolipid antigens that exist in patients' serum in the form of mucin. Their expression is directly related to the development and progression of advanced gastric cancer [17]. Herein, the eligible patients given S-1 therapy plus apatinib showed significantly lower levels of serum CEA, CA199, and CA125 versus those receiving S-1 therapy, suggesting that apatinib plus S-1 therapy can significantly reduce tumor marker expression in patients with advanced gastric cancer. The reason may be that apatinib inhibits tumor tissue cell proliferation and angiogenesis, thereby improving serum tumor marker levels [18]. Recent studies have found that cytokines are closely associated with tumor development as well as invasion, such as the *T* helper cells (Th) being divided into two subpopulations, Th1 and Th2, under the stimulation of different antigens. The Th1 subpopulation mainly secretes IFN-*γ* and IL-2 to mediate the immune function of cells [19], and the Th2 subpopulation mainly secretes cytokines such as IL-4, IL-6, and IL-10 to mediate the immune function of body fluids. The antitumor effect of the organism is mainly mediated by cellular immune function, and the decrease in the secretion of IFN-*γ* and IL-2 due to the impaired cellular immune function of the patient's organism predisposes to the development of tumors [20]. In the present study, S-1 therapy plus apatinib outperformed the single therapy of S-1 therapy in mitigating the levels of IFN-*γ*, TNF-*α*, IL-4, and IL-10, indicating that apatinib plus S-1 can effectively improve the degree of Th1 and Th2 drift in the patient's body, which consequently enhances the cytokine levels in patients with advanced gastric cancer [21].

The article "Efficacy of Apatinib plus S-1 Therapy in the Treatment of Advanced Gastric Cancer Patients and the Effect on the Levels of Tumor Markers and Th1 and Th2-Like Cytokines" was retracted in 2023. Reasons: signs of a paper mill; compromised peer review; unreliable results or conclusions.

The rectal administration of Chinese herbal medicines can avoid the bitter-cold defeat of the stomach of heat-clearing, dampness-drying, and detoxifying drugs, reduce the first-pass effect of the liver on the drugs, reduce the stimulation of the gastrointestinal mucosa, and act directly on the lesion, with faster absorption of the active ingredients of the drugs than internal drugs and no obvious toxic side effects. Intrarectal administration of Yuxianfang can regulate the balance of Th1 and Th2 cells by upregulating the expression of anti-inflammatory factors IL-10 and TGF-*β* and downregulating the expression of proinflammatory factors IFN-*γ* and TNF-*α*, thus alleviating the inflammatory response, which offers a treatment alternative.

## 6. Conclusion

The efficacy of apatinib plus S-1 therapy showed better improvement in lowering the serum tumor marker levels and ameliorating the Th1 and Th2-like cytokine levels versus S-1 therapy alone, so it is worthy of clinical application. The limitations of this study lie in the absence of long-term follow-up and the absence of studies on the drug resistance of patients. Future multicenter, randomized, prospective studies will be conducted with long-term follow-up to obtain more reliable clinical data.

The article "Efficacy of Apatinib plus S-1 Therapy in the Treatment of Advanced Gastric Cancer Patients and the Effect on the Levels of Tumor Markers and Th1 and Th2-Like Cytokines" was retracted in 2023. Reasons: signs of a paper mill; compromised peer review; unreliable results or conclusions.

## Figures and Tables

**Table 1:** Comparison of baseline data (*n* (%)).

	Observation group (*n* = 50)	Experimental group (*n* = 50)	*t* or *X*^2^	*P*
Gender			0.047	0.829
Male	34	35		
Female	16	15		
Mean age (year)	58.72 ± 6.54	58.89 ± 6.60	−0.129	0.898
Mean duration of disease (year)	3.72 ± 1.26	3.88 ± 1.31	−0.622	0.535
TNF stages			0.043	0.836
III	32	31		
IV	18	19		
Pathological types			0.047	0.829
Low differentiation	34	35		
Medium differentiation	16	15		

**Table 2:** Comparison of clinical efficacy (*n* (%)).

	Observation group (*n* = 50)	Experimental group (*n* = 50)	*X* ^2^	*P*
CR	10	19		
PR	15	21		
SD	14	7		
PD	11	3		
Total efficacy (%)	25 (50%)	40 (80%)	9.89	0.002

**Table 3:** Comparison of serum tumor marker levels ($\bar{\text{x}}$ ± *s*).

Groups	*n*	CEA (ng/mL)		CA199 (U/mL)		CA125 (U/mL)	
		Before chemotherapy	After chemotherapy	Before chemotherapy	After chemotherapy	Before chemotherapy	After chemotherapy
Observation group	50	38.52 ± 8.13	15.87 ± 3.92	74.19 ± 15.12	38.39 ± 8.51	70.27 ± 14.21	32.35 ± 7.64
Experimental group	50	38.28 ± 8.06	10.34 ± 2.61	74.35 ± 15.14	29.14 ± 6.08	70.31 ± 14.18	24.28 ± 5.09
*t*	—	0.148	8.303	-0.053	6.254	−0.014	6.216
*P*	—	0.883	＜0.001	0.958	＜0.001	0.989	＜0.001

**Table 4:** Comparison of Th1 and Th2-like cytokine levels ($\bar{\text{x}}$ ± *s*).

Groups	*n*	IFN-*γ*		TNF-*α*		IL-4		IL-10	
		Before chemotherapy	After chemotherapy	Before chemotherapy	After chemotherapy	Before chemotherapy	After chemotherapy	Before chemotherapy	After chemotherapy
Observation group	50	8.15 ± 2.07	12.28 ± 3.92	5.09 ± 1.22	6.71 ± 1.77	9.69 ± 2.85	5.17 ± 1.24	24.97 ± 7.50	13.49 ± 4.12
Experimental group	50	8.28 ± 2.11	15.39 ± 4.53	5.10 ± 1.14	8.12 ± 2.06	9.71 ± 2.79	3.77 ± 1.09	24.86 ± 7.39	9.78 ± 2.88
*t*	—	−0.311	−3.671	−0.042	−3.671	−0.035	5.996	0.074	5.219
*P*	—	0.756	＜0.001	0.967	＜0.001	0.972	＜0.001	0.941	＜0.001

**Table 5:** Comparison of adverse events.

Groups	*n*	Nausea and vomiting	Diarrhea	Weakness	Neutropenia	Thrombocytopenia	Hand-foot syndrome
Observation group	50	3	2	2	3	1	1
Experimental group	50	4	2	3	3	3	3
*X* ^2^		1.321	2.364	4.556	3.364	2.354	5.996
*P*		0.564	0.365	0.245	0.321	0.333	0.142

## Data Availability

The datasets used during the present study are available from the corresponding author upon request.

## References

[1] Ghweil A. A., Osman H. A., Hassan M. H. (2020). Validity of serum amyloid A and HMGB1 as biomarkers for early diagnosis of gastric cancer. *Cancer Management and Research*.

The article "Efficacy of Apatinib plus S-1 Therapy in the Treatment of Advanced Gastric Cancer Patients and the Effect on the Levels of Tumor Markers and Th1 and Th2-Like Cytokines" was retracted in 2023. Reasons: signs of a paper mill; compromised peer review; unreliable results or conclusions.

[2] Huang C., Liu H., Hu Y. (2022). Laparoscopic vs open distal gastrectomy for locally advanced gastric cancer. *JAMA Surgery*.

[3] Jeong S., Oh M. J., Kim U., Lee J., Kim J.-H., An H. J. (2020). Glycosylation of serum haptoglobin as a marker of gastric cancer: an overview for clinicians. *Expert Review of Proteomics*.

[4] Zhang Y., Zhu C., Lu X. (2019). [Advances in serum biomarkers for early diagnosis of gastric cancer]. *Zhejiang Da Xue Xue Bao Yi Xue Ban*.

[5] Lan C., Shen J., Wang Y. (2020). Camrelizumab plus apatinib in patients with advanced cervical cancer (clap): a multicenter, open-label, single-arm, phase II trial. *Journal of Clinical Oncology*.

[6] Zhao H., Yao W., Min X. (2021). Apatinib plus gefitinib as first-line treatment in advanced EGFR-mutant NSCLC: the phase III ACTIVE study (CTONG1706). *Journal of Thoracic Oncology*.

[7] Li Y., Sun H., Guan J., Ji T., Wang X. (2019). Serum microRNA-381: a potential marker for early diagnosis of gastric cancer. *Yonsei Medical Journal*.

[8] Meng X., Wang H., Zhao J. (2020). Apatinib inhibits cell proliferation and induces autophagy in human papillary thyroid carcinoma via the PI3K/Akt/mTOR signaling pathway. *Frontiers in Oncology*.

[9] Mizukami T., Piao Y. (2021). Role of nutritional care and general guidance for patients with advanced or metastatic gastric cancer. *Future Oncology*.

[10] Park S., Nam C. M., Kim S.-G., Mun J. E., Rha S. Y., Chung H. C. (2021). Comparative efficacy and tolerability of third-line treatments for advanced gastric cancer: a systematic review with Bayesian network meta-analysis. *European Journal of Cancer*.

[11] Peng Z., Wei J., Wang F. (2021). Camrelizumab combined with chemotherapy followed by camrelizumab plus apatinib as first-line therapy for advanced gastric or gastroesophageal junction adenocarcinoma. *Clinical Cancer Research*.

[12] Qin S., Li Q., Gu S. (2021). Apatinib as second-line or later therapy in patients with advanced hepatocellular carcinoma (AHELP): a multicentre, double-blind, randomised, placebo-controlled, phase 3 trial. *The Lancet Gastroenterology & Hepatology*.

[13] Seeneevassen L., Bessède E., Mégraud F., Lehours P., Dubus P., Varon C. (2021). Gastric cancer: advances in carcinogenesis research and new therapeutic strategies. *International Journal of Molecular Sciences*.

[14] Siebenhüner A. R., De Dosso S., Helbling D., Astaras C. (2021). Advanced gastric cancer: current treatment landscape and a future outlook for sequential and personalized guide: Swiss expert statement article. *Oncology research and treatment*.

[15] Tokunaga M., Sato Y., Nakagawa M. (2020). Perioperative chemotherapy for locally advanced gastric cancer in Japan: current and future perspectives. *Surgery Today*.

The article "Efficacy of Apatinib plus S-1 Therapy in the Treatment of Advanced Gastric Cancer Patients and the Effect on the Levels of Tumor Markers and Th1 and Th2-Like Cytokines" was retracted in 2023. Reasons: signs of a paper mill; compromised peer review; unreliable results or conclusions.

[16] Xie C., Zhou X., Liang C. (2021). Apatinib triggers autophagic and apoptotic cell death via VEGFR2/STAT3/PD-L1 and ROS/Nrf2/p62 signaling in lung cancer. *Journal of Experimental & Clinical Cancer Research*.

[17] Wei L., Sun J., Zhang N. (2020). Noncoding RNAs in gastric cancer: implications for drug resistance. *Molecular Cancer*.

[18] Xie L., Xu J., Sun X., Guo W. (2020). Apatinib plus camrelizumab (anti-PD1 therapy, SHR-1210) for advanced osteosarcoma (APFAO) progressing after chemotherapy: a single-arm, open-label, phase 2 trial. *Journal for immunotherapy of cancer*.

[19] Xu J., Shen J., Gu S. (2021). Camrelizumab in combination with apatinib in patients with advanced hepatocellular carcinoma (rescue): a nonrandomized, open-label, phase II trial. *Clinical Cancer Research*.

[20] Yang Q.-K., Chen T., Wang S.-Q., Zhang X.-J., Yao Z.-X. (2020). Apatinib as targeted therapy for advanced bone and soft tissue sarcoma: a dilemma of reversing multidrug resistance while suffering drug resistance itself. *Angiogenesis*.

[21] Yang S., He X., Liu Y. (2019). Prognostic significance of serum uric acid and gamma-glutamyltransferase in patients with advanced gastric cancer. *Disease Markers*.

